The article "Comparison of Clinical Pregnancy Outcomes after Fresh and Frozen Embryo Transfer" was retracted in 2023. Reasons: signs of a paper mill; compromised peer review; unreliable results or conclusions.

# Comparison of Clinical Pregnancy Outcomes after Fresh and Frozen Embryo Transfer

**DOI:** 10.1155/2022/6498356

**Published:** 2022-10-03

**Authors:** Hui Yu, Yuehong Zhang, Mei Han

**Affiliations:** Department of Gynecology and Obstetrics, Tongzhou District Maternal and Child Health Hospital, Beijing City 101199, China

## Abstract

**Objectives:**

To analyze the clinical outcomes of the patients who underwent fresh or frozen embryo transfer, as well as the neonatal outcomes.

**Methods:**

We conducted a retrospective analysis of women who underwent *in vitro* fertilization with fresh and frozen embryo transfer from January 2019 to January 2021. All of the included embryo transfers resulted in live births at ≥28 weeks of gestation. All of the patients were divided into two groups according to the assisted reproductive technique that was used (fresh embryo transfer group (*n* = 101) and frozen embryo transfer group (*n* = 125)). Both groups were divided into subgroups based on a maternal age of ≥35 years. *Result(s)*. Between the two groups, only the cesarean section rate was higher in the frozen transfer group, while no differences were shown for other outcomes. There were significant differences in the gestational hypertension and postpartum hemorrhage rates based on the subgroup comparison. No significant differences were detected in the offspring.

**Conclusions:**

Comparing fresh and frozen embryo transfers did not reveal any significant superiority. Venerable age exerts an apparent influence on pregnancy complications. Frozen embryo transfer is not always the best choice.

## 1. Introduction

The world's first baby conceived via *in vitro* fertilization (IVF) was born in England in July 1978, marking the new era of assisted reproductive technologies. The first baby conceived via IVF in China was born in Beijing in 1988 at Peking University Third Hospital. Since then, China has recorded an impressive prosperity of assisted reproductive technologies. Statistics show that there are >50 million infertile women in China today, accounting for 15% of all women of childbearing age [1]. This number continues to grow. Assisted reproductive technologies offers new hope for more and more infertile couples and also has a tremendous impact on social development in China. At present, IVF and embryo transfer (IVF-ET) technology is the primary treatment for infertility. Fresh or frozen embryo transfer is an integral part of this technology. The advantages, disadvantages, and indications for IVF-ET, however, remain controversial topics. In earlier years, the fertility, pregnancy loss, and live birth rates received priority attention. As assisted reproductive technologies have matured, the focus has shifted from live births to improved birth outcomes. The embryo quality and perinatal complications in pregnant women and newborns are the new priorities. Some international institutions have proposed replacing fresh embryo transfer entirely with frozen embryo transfer according to the analysis of massive amounts of data. So, the question is: Are pregnancy outcomes better with frozen embryo transfer than fresh embryo transfer? We collected data on maternal outcomes during the perinatal period and neonatal complications after IVF and obstetric examinations at our hospital from 2019 to 2021. The maternal and perinatal outcomes were compared after fresh and frozen embryo transfer as to identify the strengths and weaknesses of each ET method.

## 2. Materials and Method

### 2.1. General Information

We collected and analyzed the data of patients and newborns after IVF-ET at our hospital from January 2019 to January 2021. The inclusion criteria were as follows: (1) pregnant after frozen or fresh embryo transfer; and (2) gestational age ≥ 28 weeks at the time of delivery. The exclusion criteria were as follows: (1) the method of assisted reproduction not recorded and (2) medical complications, such as diabetes and hypertension, which might affect pregnancy outcomes. The patients were classified into fresh or frozen embryo transfer groups depending on the assisted reproductive technologies used.

### 2.2. Method

The baseline maternal characteristics, pregnancy complications, pregnancy outcomes, and perinatal outcomes of the newborns were collected. The maternal age, type of infertility, pregnancy complications, delivery mode, and obstetric labor complications were analyzed. The newborn gender, birth weight, perinatal complications, and birth defects were analyzed. Special emphasis was placed on obstetric labor and neonatal complications.

### 2.3. Statistical Analysis

All statistical analyses were performed using SPSS26.0 software. The normality test was applied to the measurement data of the two groups. The maternal ages of both groups were followed a normal distribution. If the measurement data obeyed a normal distribution, the means were expressed as $\bar{x}\pm s$ and compared using a two-sample independent t-test. Counts are expressed as [*n* (%)] and analyzed using the *χ*^2^ test. A significant difference was indicated by a *P* < 0.05.

## 3. Results

### 3.1. Comparison of Baseline Maternal Characteristics

One hundred and twenty-five patients underwent fresh embryo transfer, and 101 patients underwent frozen embryo transfer.

The women receiving fresh and frozen embryo transfers did not differ significantly in average age and the rate of multifetal pregnancies (*P* > 0.05). A comparison was made between different types of infertility. Patients with primary and secondary infertility between the fresh and frozen embryo transfer groups differed significantly (*P* < 0.05; Table 1).

### 3.2. Comparison of Maternal Pregnancy Outcomes

The incidence of several pregnancy complications was not significantly different between the patients in the two groups (*P* > 0.05). The pregnancy complications that were analyzed included the following: gestational diabetes, gestational hypertension, premature rupture of membranes, chorioamnionitis, c-section, postpartum bleeding, fetal distress, abnormal amniotic fluid volume, abnormal placental location, and preterm birth. The two groups differed significantly in cesarean section rate (*P* < 0.05; Table 2).

### 3.3. Comparison of Neonatal Outcomes between the Two Groups

The gender ratio was comparable between the two groups. There were no significant differences in the average birth weight between the two groups (*P* > 0.05). No significant differences were observed in the incidence of perinatal complications of the newborns between the two groups, including macrosomia, very low birth weight infants, neonatal hyperbilirubinemia, and other birth defects (*P* > 0.05; Table 3).

### 3.4. Intragroup Comparison of Pregnancy Outcomes in Young Women and Women of Advanced Maternal Age

Women receiving fresh embryo transfer were further divided into two subgroups (young women and women of advanced maternal age). We observed a significant increase in the incidence of gestational hypertension and postpartum bleeding in the advanced maternal age subgroup compared with the young maternal age group (*P* < 0.05). There was no significant difference in the incidence of gestational diabetes, premature rupture of membranes, chorioamnionitis, caesarean section rate, fetal distress, abnormal amniotic fluid volume, abnormal placental location, and preterm birth (*P* > 0.05; Table 4). We noted a significant increase in the cesarean section rate between the advanced and young maternal age groups (*P* < 0.05) who underwent frozen embryo transfer. There was no significant difference in the incidence of other pregnancy complications among the patients (*P* > 0.05; Table 5).

### 3.5. Intragroup Comparison of Baseline Neonatal Characteristics between the Young Mother and Advanced Maternal Age Subgroups

There were no significant differences in gender ratio, average birth weight, or the incidence of perinatal complications among the newborns between the two subgroups, including macrosomia, very low birth weight infants, neonatal hyperbilirubinemia, and other birth defects (*P* > 0.05; Tables 6 and 7).

## 4. Discussion

IVF-ET is an assisted reproductive technique that currently has extensive applications. Along with continued technologic progress and experience in assisted reproductive technologies, a growing number of medical institutions now favor frozen embryo transfer over fresh embryo transfer to reduce ovarian hyperstimulation and increase the cumulative pregnancy rate. There are even strong advocates for a freeze-only strategy. Frozen embryo transfer can more closely mimic the physiologic state during embryo implantation [2]. Nevertheless, the long-term maternal and neonatal safety requires further investigation. As the number of babies born following IVF continues to increase, the research and surveys focusing on perinatal outcomes among patients and newborns have been expanded. A comparative assessment of fresh and frozen embryo transfers is also underway.

We compared maternal outcomes during the perinatal period between fresh and frozen embryo transfers and arrived at the following conclusions. The incidence of pregnancy complications was not significantly different between patients in the two groups (*P* ≥ 0.05), including gestational diabetes, gestational hypertension, premature rupture of membranes, chorioamnionitis, postpartum bleeding, fetal distress, abnormal amniotic fluid volume, abnormal placental location, and preterm birth; however, patients with primary and secondary infertility between the fresh and frozen embryo transfer groups differed significantly (*P* = 0.001, <0.05). The two groups differed significantly with respect to the c-section rate (*P* = 0.041, <0.05). There were no significant differences in gender ratio, average birth weight, or the incidence of perinatal complications among the newborns between the two groups, including macrosomia, very low birth weight infants, neonatal hyperbilirubinemia, and other birth defects (*P* ≥ 0.05). Based on our literature review, the conclusions drawn from the comparison of maternal outcomes in the perinatal period between fresh and frozen embryo transfers continue to attract controversy. In a retrospective study, Guo et al. [3] included 1516 parturients who delivered singletons, which showed that frozen embryo transfer was associated with a higher risk of placenta previa, postpartum bleeding, and placental adhesion compared to fresh embryo transfer (the differences all being statistically significant). Frozen embryo transfer was an independent risk factor for postpartum bleeding and placental adhesion. Xiong et al. [4] conducted a retrospective analysis that indicated a correlation between gestational hypertension and intracytoplasmic sperm injection; however, frozen embryo transfer did not increase the risk of gestational hypertension. According to other studies [5–7], frozen embryo transfer reduced the risks of ovarian hyperstimulation, ectopic pregnancy, gestational hypertension, placental abruption, and ischemic placental disease. In addition, the incidence of preterm birth and low birth weight infants was lower with frozen embryo transfer than fresh embryo transfer, although the risk of macrosomia increased. Chen et al. [8] studied the perinatal outcomes in 120 dizygotic twins conceived via IVF and reported comparable overall outcomes in twin pregnancies after fresh and frozen embryo transfer. No significant differences were observed in a comparison of several perinatal complications. Moreover, the neonatal complications in the postnatal period were compared and no significant differences between the two groups were reported.

Ainsworth et al. [9] conducted a survey involving the body weight of 136 newborns conceived via IVF, including 87 newborns via fresh embryo transfer and 49 newborns via frozen embryo transfer. The newborns conceived via different techniques did not differ significantly in birth weight, body length, or head circumference (*P* < 0.05). The newborns were followed for at least 18 months or until 5 years of age if conditions permitted. The results showed that the differences between the two groups of newborns diminished after correction for the newborn body length, head circumference, and gender, as well as gestational age and maternal health. No significant differences were observed in the subsequent growth of the newborns. Thus, it was concluded that fresh and frozen embryo transfer did not differ considerably in the impact on body weight from birth-to-childhood. Magnus et al. [10] believed that the newborns conceived via IVF had lower body weight and shorter body length compared with naturally conceived newborns. In contrast, the newborns conceived via frozen embryo transfer had comparable body weight and body length as the naturally conceived newborns. Eighteen months after birth, however, newborns artificially conceived had compensatory growth and differed very little from the naturally conceived newborns during subsequent observations. According to other studies [11–13], the body weight of newborns conceived by fresh and frozen embryo transfer differ. One possible reason is that frozen embryo transfer affects the newborn birth weight and height at the level of embryonic epigenetics. The maternal high levels of estrogen during fresh embryo transfer negatively influence fetal growth and development by inhibiting invasion of spiral arteries, impairing placental blood flow, and causing placental hypoperfusion. van Duijn et al. [14] contended that the birth weight was lower after fresh embryo transfer; however, most of the abovementioned studies only provided a rough estimate, and there are many factors at play when it comes to the influence on birth weight. A longitudinal follow-up study is needed for newborns conceived via different methods of assisted reproduction to better identify the correlated factors.

Depending on the maternal age at the time delivery, the patients were divided into young (<35 years of age) and advanced age subgroups (≥35 years of age). An intragroup comparison showed a significant difference in the incidence of gestational hypertension and postpartum bleeding between the young and advanced age subgroups after fresh embryo transfer (*P* < 0.05). There was a significant difference in the cesarean section rate between the young and advanced age subgroups after frozen embryo transfer (*P* < 0.05); however, no significant difference was observed between the young and advanced age subgroups after fresh embryo transfer or between the young and advanced age subgroups after frozen embryo transfer. There are a large number of studies showing that gestational hypertension is influenced by a multiplicity of factors, including age, genetics, gravidity and parity, and singleton or multiple pregnancies [15]. Advanced age is an independent risk factor for adverse maternal and neonatal outcomes [16]. In addition, manipulations during embryo transfer [17] may impair endometrial receptivity, which further affects the invasive capability of placental trophoblast cells, inducing placenta-derived diseases. Women of advanced age usually have decreased vascular elasticity and changing hormone levels, thus increasing the risk of vascular sclerosis. Uterine blood vessels may be also affected, increasing the risk of associated complications [18]. Moreover, a large number of clinical epidemiologic surveys have shown that gestational hypertension may alter coagulation function or even lead to coagulation dysfunction, increasing the risk of postpartum bleeding. In parturients of advanced age, the incidence of uterine inertia increases considerably. Considering the influence of a myriad of factors, several pregnancy complications may interact with each other. With respect to the difference in cesarean section rate after fresh and frozen embryo transfer, we believe that the parturients undergoing frozen embryo transfer and their relatives are more concerned about the potential risks associated with natural birth. These patients are usually of an older age and have already faced longer IVF cycles and greater economic burden. For these reasons, a larger proportion of patients undergoing frozen embryo transfer prefer cesarean section than those undergoing fresh embryo transfer. Cesarean section shortens the labor process and avoids compression of the newborn passing through the birth canal. In addition, the possibility of fetal distress and relevant complications decreases with cesarean section.

According to the data, either fresh embryo transfer or frozen embryo transfer, advanced maternal age shows different degrees of influence. For those who accepted fresh embryo transfer, the incidence of hypertensive disorders during pregnancy and postpartum hemorrhage rates significantly increased, while for those who accepted frozen embryo transfer, the c-section rate significantly increased. Those increases in complication rate may lead to different maternal and fetal outcomes [19–21]. Combined with the clinical situation, we could carry out production inspection plan including some individual treatments for those patients with high risks, so as to minimize the adverse effects. Referring to the control of cesarean section rate, we could fully inform patients the advantages and disadvantages of both modes of delivery, appropriately encourage the patients to have a trial labor, and strengthen monitoring during labor, so as to lower the complication rates.

To conclude, we suggest the need for individualized decision-making in IVF based on the patients' specific conditions. There should be a comprehensive consideration of the pros and cons of each technique to avoid complications and safeguard maternal and neonatal health. Celada et al. [22] offered a detailed description of the pros, cons, and current indications of the freeze-only strategy. As we have pointed out, the choice of IVF technique should be based on patients' individual situation and a sufficient consideration about the benefits and risks of the technique chosen. The long-term outcomes of IVF with fresh or frozen embryo transfer remain to be further investigated. The 2018 Data Report on assisted reproductive technologies released by the Chinese Society of Reproductive Medicine in 2021 [23] has pointed out that the prevalence of freeze-only strategy began to increase every year since 2016. The reasons for this finding are two-fold: first, the importance of uterine conditions in IVF is overemphasized; and second, the freeze-only strategy reduces the incidence of ovarian hyperstimulation. In the face of increasingly extended applicability of the freeze-only strategy, we should pay due attention to the prolonged IVF cycles and increased economic burden for patients, as well as the potential alteration of embryonic epigenetics and the fetal safety problem. Based on our data, it is easy to detect dramatic differences in the incidence of pregnancy complications; however, the differences were not of statistical significance after an in-depth analysis. Given the small sample size and the limitations of the present study, the conclusions should be corroborated through additional cases of IVF and valid analyses.

## Figures and Tables

**Table 1:** Comparison of baseline maternal characteristics between patients undergoing fresh and frozen embryo transfer [*n* (%)].

Baseline	Fresh embryo transfer (*n* = 125)	Frozen embryo transfer (*n* = 101)	*P* value
Average age (year)	32.53 ± 3.80	33.13 ± 4.87	0.311
Different types of infertility	—	—	—
Primary infertility [*n* (%)]	78 (62.4%)	64 (63.37%)	0.001
Secondary infertility [*n* (%)]	47 (37.6%)	37 (36.63%)	0.001
Twin pregnancy [*n* (%)]	26 (20.8%)	17 (16.83%)	0.450

**Table 2:** Comparison of maternal pregnancy outcomes after fresh and frozen embryo transfer [*n* (%)].

Pregnancy complications	Fresh embryo transfer (*n* = 125)	Frozen embryo transfer (*n* = 101)	*P* value
Gestational diabetes	47 (37.60%)	46 (45.54%)	0.228
Gestational hypertension	16 (12.80%)	10 (9.90%)	0.497
Premature rupture of membranes	39 (31.20%)	22 (21.78%)	0.113
Chorioamnionitis	7 (5.60%)	7 (6.93%)	0.680
Cesarean delivery	91 (72.80%)	85 (84.26%)	0.041
Postpartum bleeding	14 (11.20%)	12 (11.88%)	0.873
Fetal distress	8 (6.40%)	5 (4.95%)	0.642
Abnormal amniotic fluid volume	11 (8.80%)	6 (5.94%)	0.418
Abnormal placental location	6 (4.80%)	2 (1.98%)	0.260
Preterm birth	27 (21.60%)	18 (17.82%)	0.479

**Table 3:** Comparison of neonatal outcomes after fresh and frozen embryo transfer [n(%)].

Neonatal outcomes	Fresh embryo transfer (*n* = 125)	Frozen embryo transfer (*n* = 101)	*P* value
Average birth weight	3120.07 ± 561.18	3147.14 ± 621.10	0.720
Macrosomia	8 (6.40%)	10 (9.90%)	0.334
Very low birth weight infants	11 (8.80%)	9 (8.91%)	0.977
Neonatal hyperbilirubinemia	6 (4.80%)	3 (2.97%)	0.484
Other birth defects	3 (2.40%)	3 (2.97%)	0.791
Gender ratio (male/female)	76/75	55/63	0.618

**Table 4:** Comparison of pregnancy outcomes between young and advanced age subgroups after fresh embryo transfer.

Pregnancy outcomes of fresh embryo transfer	Young maternal age subgroup (*n* = 92)	Advanced maternal age subgroup (*n* = 33)	*P* value
Caesarean section	65 (70.65%)	26 (78.79%)	0.368
Gestational diabetes	32 (34.78%)	15 (45.45%)	0.278
Gestational hypertension	8 (8.70%)	8 (24.24%)	0.022
Premature rupture of membranes	29 (31.52%)	10 (30.30%)	0.897
Chorioamnionitis	7 (7.61%)	0 (0%)	0.103
Postpartum bleeding	7 (7.61%)	7 (21.21%)	0.034
Fetal distress	6 (6.52%)	2 (6.06%)	0.926
Abnormal amniotic fluid volume	10 (10.87%)	1 (3.03%)	0.315
Abnormal placental location	4 (4.35%)	2 (6.06%)	0.693
Preterm birth	20 (21.74%)	7 (21.21%)	0.855

**Table 5:** Comparison of pregnancy outcomes between young and advanced age subgroups after frozen embryo transfer.

Pregnancy outcomes of frozen embryo transfer	Young maternal age subgroup (*n* = 67)	Advanced maternal age subgroup (*n* = 34)	*P* value
Gestational diabetes	27 (40.30%)	18 (52.94%)	0.227
Gestational hypertension	8 (11.94%)	2 (5.88%)	0.335
Premature rupture of membranes	18 (26.87%)	6 (17.65%)	0.304
Chorioamnionitis	6 (8.96%)	1 (2.94%)	0.261
Caesarean section	52 (77.61%)	33 (97.06%)	0.011
Postpartum bleeding	8 (11.94%)	4 (11.76%)	0.979
Fetal distress	4 (5.97%)	2 (5.88%)	0.986
Abnormal amniotic fluid volume	3 (4.48%)	3 (8.82%)	0.383
Abnormal placental location	2 (2.99%)	0 (0%)	0.309
Preterm birth	13 (19.40%)	5 (14.71%)	0.560

**Table 6:** Comparison of neonatal outcomes between young and advanced age subgroups after fresh embryo transfer.

Neonatal outcomes of fresh embryo transfer	Young maternal age subgroup (*n* = 92)	Advanced maternal age subgroup (*n* = 33)	*P* value
Average birth weight (g)	3041.95 ± 597.08	3223.78 ± 586.26	0.108
Macrosomia	6 (6.52%)	2 (6.06%)	0.926
Very low birth weight infants	8 (8.70%)	3 (9.09%)	0.945
Neonatal hyperbilirubinemia	4 (4.35%)	2 (6.06%)	0.693
Other birth defects	3 (3.26%)	0 (0%)	0.294

**Table 7:** Comparison of neonatal outcomes between young and advanced age subgroups after frozen embryo transfer.

Neonatal outcomes of frozen embryo transfer	Young maternal age subgroup (*n* = 67)	Advanced maternal age subgroup (*n* = 34)	*P* value
Average birth weight (g)	3142.28 ± 638.05	3175.90 ± 681.60	0.791
Macrosomia	8 (11.94%)	3 (8.82%)	0.635
Very low birth weight infants	6 (8.96%)	3 (8.82%)	0.982
Neonatal hyperbilirubinemia	3 (4.48%)	0 (0%)	0.210
Other birth defects	2 (2.99%)	1 (2.94%)	0.990

## Data Availability

All data, models, and code generated or used during the study appear in the submitted article.
